The article "Early warning of telecom enterprise customer churn based on ensemble learning" was published in 2023. Journal: PLoS One.

# Early warning of telecom enterprise customer churn based on ensemble learning

**DOI:** 10.1371/journal.pone.0292466

**Published:** 2023-10-11

**Authors:** Yancong Zhou, Wenyue Chen, Xiaochen Sun, Dandan Yang

**Affiliations:** 1 School of Information Engineering, Tianjin University of Commerce, Tianjin, China; 2 College of Management and Economics, Tianjin University, Tianjin, China; XJTLU: Xi’an Jiaotong-Liverpool University, CHINA

## Abstract

Analyzing customers’ characteristics and giving the early warning of customer churn based on machine learning algorithms, can help enterprises provide targeted marketing strategies and personalized services, and save a lot of operating costs. Data cleaning, oversampling, data standardization and other preprocessing operations are done on 900,000 telecom customer personal characteristics and historical behavior data set based on Python language. Appropriate model parameters were selected to build BPNN (Back Propagation Neural Network). Random Forest (RF) and Adaboost, the two classic ensemble learning models were introduced, and the Adaboost dual-ensemble learning model with RF as the base learner was put forward. The four models and the other four classical machine learning models-decision tree, naive Bayes, K-Nearest Neighbor (KNN), Support Vector Machine (SVM) were utilized respectively to analyze the customer churn data. The results show that the four models have better performance in terms of recall rate, precision rate, F1 score and other indicators, and the RF-Adaboost dual-ensemble model has the best performance. Among them, the recall rates of BPNN, RF, Adaboost and RF-Adaboost dual-ensemble model on positive samples are respectively 79%, 90%, 89%,93%, the precision rates are 97%, 99%, 98%, 99%, and the F1 scores are 87%, 95%, 94%, 96%. The RF-Adaboost dual-ensemble model has the best performance, and the three indicators are 10%, 1%, and 6% higher than the reference. The prediction results of customer churn provide strong data support for telecom companies to adopt appropriate retention strategies for pre-churn customers and reduce customer churn.

## Introduction

In the current environment where domestic mobile communication users are close to China’s total population and the three major telecom operators share the entire telecommunications market equally. The remaining customer market is becoming more and more sparse, and the gap between the maintenance costs of new and old customers is becoming more and more obvious. According to the American Marketing Association’s Customer Satisfaction Handbook, it costs five times as much to attract a new customer as to maintain an existing one. Therefore, the strategic focus of communication operators should change from ‘product-centric’ to ‘customer-centric’. Telecom operators possess a huge user group, which means it is unrealistic to pay attention to the demands of each customer. If the company can accurately predict the future loss of customers, it can not only save a lot of human, material and financial resources, but also implement targeted retention strategy, improve customer stickiness, and better explore the high sustainable profit and low maintenance cost brought by old customers, thereby improve the core competitiveness of the enterprise.

The article "Early warning of telecom enterprise customer churn based on ensemble learning" was published in 2023. Journal: PLoS One.

With the increasing popularity of machine learning, machine learning models are favored in the field of customer churn. Machine learning models can be roughly divided into two categories: basic learning models and ensemble learning models. Basic learning models include linear models, logistic regression, decision trees, Artificial Neural Networks (ANNs), etc. The ensemble learning models are based on basic learners (i.e. weak learners), which are combined into a strong learning model through specific ensemble rules. Ensemble learning refers to the combination of multiple models to obtain better results, that is, multiple weak learners are combined into a strong learner, so that the integrated model has stronger generalization ability. According to the different integration methods, it can be divided into two categories: Boosting and Bagging. Common ensemble rules include Adaboost (Adaptive Boosting algorithm), a typical representative of the Boosting, and RF, a derivative algorithm of the Bagging.

At present, the research focus in the field of machine learning has gradually shifted from improving basic learners to studying the ensemble strategy of multiple basic learners. Ji Huijie selected XGBoost, RF, improved logistic regression model based on recursive feature elimination, and embedded Adaboost model in predicting telecom customer churn [1]. The XGBoost algorithm with an F1 score of 70.98% is better than the other three. Ren Lulu also uses Adaboost, RF, and XGBoost in the field of customer churn prediction in auto 4S stores. Her research proves that the prediction performance of the Adaboost model is higher than other integrated learners [2]. Li Ying also selected basic and ensemble learners to analyze the loss of users of the course live broadcast platform, including decision trees, XGBoost, and RF [3]. The results show that XGBoost and RF in the ensemble model have their own strengths in precision and recall. But both outperform the base learner.

In addition, many current researches choose to try to combine ensemble learning models, and they all achieve better prediction results in specific subjects. Chen Peng predicted customer churn based on the hotel customer visit data publicly released by Ctrip, and established five models: logistic regression, XGBoost, RF, Supported Vector Machine, and Naive Bayes [4]. The Naive Bayes was removed due to poor evaluation results, and the other four models were ensembled through Stacking as the optimal hotel customer churn prediction model with an F1 score of 94.8%, which is 1.6% higher than the RF with the best prediction effect. Li Jiahao also used Stacking-based Adaboost and RF ensemble model—LRA model in the research on employee turnover prediction, which greatly improved the accuracy and robustness of the original learner [5]. Zhang Mengdi’s research on the churn of bank credit card customers shows that using the Stacking ensemble learning method to integrate the two single models of logistic regression and XGBoost, the combined model shows better prediction performance [6]. According to these studies, when the performance of the model’s performance is difficult to improve, it can be improved by building a combined model. Therefore, under the research trend of quadratic combination of ensemble models, this paper attempts to combine RF and Adaboost quadratically into a dual-ensemble model to predict customer churn. From the perspective of bias-variance decomposition, the Bagging method represented by RF model mainly focuses on reducing variance and has good anti-noise ability; the Boosting method represented by Adaboost model mainly focuses on reducing bias, and a strong ensemble learner can also be constructed based on learners with weak generalization performance [7]. So, this paper attempts to propose the RF-Adaboost dual-ensemble model to give full play to the advantages of the two models, hoping to get better experimental results.

The article "Early warning of telecom enterprise customer churn based on ensemble learning" was published in 2023. Journal: PLoS One.

The customer personal information and historical behavior data sets of telecom operators are studied, and three classic learning models: BPNN, RF, and Adaboost are selected. And the RF-Adaboost dual-ensemble model based on RF learner for customer churn prediction is proposed. The code is based on the Python language, and the Jupyter Notebook development tool completes the code writing and running. The evaluation is given according to the prediction results of the training model, and the average precision rate, recall rate, F1 score and the according weighted value are selected as evaluation indicators. Additionally, the prediction results are displayed intuitively by the ROC curve. The learning model with the best recall rate is selected for customer churn early warning.

## Data and data preprocessing

### Data sources

In this paper, the real user data from a certain operator is used for model training and analysis. The operator’s customer original data set shows the personal attributes and behavior data of different users within three months, a total of 900,000 pieces, and each data record contains 35 feature attributes, including user ID, contract status, online time, call status, traffic usage, etc. The last column (i.e. the dependent variable) is the identification of whether the user has lost or not. 0 represents a negative sample that has not been lost, and 1 represents a positive sample that has been lost.

### Data preprocessing

To different attribute values and data types, data cleaning, imbalance processing, data standardization and other preprocessing operations on a certain operator’s customer personal characteristics and historical behavior data set are conducted. Initially, irrelevant features, redundant features, non-numeric features are deleted and transformed. Then missing values, outliers, and duplicate values are processed. SMOTE (Synthetic Minority Oversampling Technique) is used for the imbalance of positive and negative samples in the dataset. Finally, preprocessed data is standardized and effectively divided into the training set and the test set. The original operator customer data set contains 35 features and 900,000 samples, of which the ratio of positive and negative samples is 1:30. After data preprocessing and merging, 14 features and 386,269 samples are remained, and the ratio of positive and negative samples is 2:5.

Regarding the problem of data imbalance, Nathalie Japkowicz proved as early as 2002 that most machine learning models such as neural network and RF cannot exert normal predictive ability when the difference between the number of positive and negative samples is large [8]. According to the analysis of such data imbalance problem, the current operator customer data set has a total of 285,287 user data after data preprocessing, of which 275,907 are online users (i.e. negative samples) and 9,380 are offline users. The ratio of majority to minority samples is about 30:1. Therefore, the SMOTE method is used to oversample the data, and the sampling strategy parameter sampling_strategy is selected to be 0.4, that is, the ratio of positive and negative samples after sampling is 4:10. The data set obtained 386,269 samples, of which the number of negative samples is still 275,907, while the number of positive samples has increased to 110,362.

## The customer churn prediction model based on machine learning

### Prediction model based on BPNN

#### Basic principle and structure of BPNN

BPNN is a feed-forward neural network to enhance the classification and recognition capabilities of the network and solve nonlinear problems. It combines the error back propagation algorithm discovered by David Runelhart et al. in the 1980s. The basic idea is Gradient descent, which uses gradient search techniques to minimize the mean-square error between the network output value and the expected value. In the field of binary classification, the application of BPNN has been relatively mature and extensive. Shi Danlei established a BPNN in the problem of bank customer churn prediction, and proved that through continuous iterative training, the accuracy rate kept increasing and the loss value continued to decrease [9]. Farzaneh Mohammadi used a single-layer feed-forward neural network to achieve a more stable model than logistic regression to characterize COVID-19 infected patients in local areas of Iran [10]. Li Xiangqing et al. proved that the prediction accuracy of deep neural network for customer churn is higher than that of SVM, logistic regression, RF, and Adaboost [11]. As the most widely used form of neural network at present, BPNN has strong self-learning and self-adaptive capabilities, and can automatically search for reasonable rules between input and output through data sets, and feed back into network weights for memory. In addition, it shows good generalization and fault tolerance for various problems in different fields. Therefore, this paper selects BPNN as one of the prediction models of customer churn.

The article "Early warning of telecom enterprise customer churn based on ensemble learning" was published in 2023. Journal: PLoS One.

The BPNN model includes two processes: forward propagation and error back propagation:

(1) forward propagation—The process is the same as the general feedforward neural network. The input signal is weighted and summed by the weight value of the intermediate hidden layer, and then the activation function is input to obtain the result and output to the next layer. Eq (1) can be used to express the i-th layer:
$$h_{out}^{i}=f_{actv}^{i}(h_{in}^{i}w^{i}+\theta^{i})$$ (1)
  where ***h***_***out***_ is the output matrix, ***h***_***in***_ is the input matrix, ***w*** is the weight matrix, ***θ*** is the threshold vector, and ***f***_***actv***_ is the activation function.
(2) Error back propagation—After getting the output, BPNN will calculate the error between the output value and the expected value through a specific regression loss function, generally using the L2-loss mean-square error function, which is shown in Formula (2):
$$E=\frac{1}{2}{\left(O-L\right)}^{2}$$ (2)
  where ***E*** is the error value, ***O*** is the output value matrix, and ***L*** is the expected value matrix. Then, the weight ***w*** and the threshold ***θ*** are updated by the gradient descent method, and the formula is shown in Formula (3):
$$\Delta Param=\eta \frac{\partial E}{\partial Param}$$ (3)
  where ***Param*** is the weight or threshold to be updated, ***E*** is the error obtained by the loss function, and ***η*** is the learning rate. If the learning rate is too large, the optimal solution may be exceeded, and if it is too small, the efficiency of the algorithm may be reduced. The above is an Epoch of the neural network. When the model judges that the error meets the accuracy requirements, the iterative training ends.

The article "Early warning of telecom enterprise customer churn based on ensemble learning" was published in 2023. Journal: PLoS One.

#### BPNN model design and implementation

The 14 feature columns in the current customer data set are used as the 14 input layer nodes of the BPNN. After processing through several hidden layers, the output layer activation function is mapped to the (0, 1) interval, and the predicted output result of 0 or 1 is obtained. Therefore, the output layer contains only a single node. The specific structure of the BPNN is shown in Fig 1:

**Fig 1:** BPNN’s structure.

The optimization of the BPNN model is the adjustment of specific parameters, such as adding hidden layers, adding single-layer neurons, increasing the maximum number of iterations, selecting different weight optimizers and activation functions, etc. In the early warning research on financial risks, Wang Ting et al. constructed a variety of BPNN models to compare the results, and found that when the number of hidden layers increased from 1 to 3, the model learning accuracy and learning rate were more obvious improvement [12]. However, as the complexity of the hidden layer network increases, the learning efficiency of a single neuron node decreases, the network convergence speed decreases, and the error increases. Therefore, this study selects the most suitable model by repeatedly adjusting the parameters of the BPNN and comparing various indicators.

The basic parameters of the BPNN model are analyzed respectively, and the following conclusions are drawn:

(1) Hidden layer structure—In the field of neural network modeling, the structure of the hidden layer is the focus of adjustment. Many studies have used two empirical formulas, and on this basis, the floating test is performed, as shown in Formulas (4) and (5):
x=2m+1 (4)
$$h=\sqrt{n+m}+a$$ (5)
  Where ***x*** is the number of hidden nodes, ***h*** is the number of hidden layers, ***m*** is the number of input layer nodes, ***n*** is the number of output layer nodes, and ***a*** is any constant between 1 and 10. It can be seen from the calculation that for the customer churn dataset in this study, the best possible structure is 4~14 hidden layers and a total of 29 hidden nodes. In this paper, it is found through experiments that appropriately increasing the hidden layer can greatly improve the prediction performance of the model. However, with the further increase of the number of layers, the training time gradually increases while the result is not improved or even slightly reduced. Among them, the best effect and the shortest time are used. The hidden layer structure is 12-16-5, including 3 layers of 33 hidden nodes, which is similar to the result calculated by the empirical formula.
(2) Weight optimizer—Among the three weight optimizers commonly used in the current research field, L-BFGS is usually used in high-dimensional data analysis research, and can only show obvious advantages when the feature dimension is high. SGD (Stochastic Gradient Descent) is to randomly optimize the loss function on a certain piece of training data to converge the parameters to the local optimum, so the accuracy decreases while the parameter update speed is accelerated. In contrast, Adam combining AdaGrad (Adaptive Gradient) and RMSProp (Root Mean Square Propagation) is one of the most popular optimizers in deep learning. Its ease of fine-tuning allows it to achieve good results quickly. It uses the same learning rate for each parameter, and adapts independently as learning through the history of gradients. Francesco Orabona, an assistant professor at Boston University, once said: "It is not Adam that is the best, but the training of the neural network to make it the best." It can be seen that Adam is one of the most suitable weight optimizers for BPNN, and the experimental results have also proved it.
(3) Activation function—Sigmoid, also known as logistic regression function, maps the input value into the (0, 1) interval. It is a popular traditional neural network activation function, but when the sample is compressed into a narrow interval with a step size of 1, it will cause the saturation of the value range. And according to the Sigmoid image, it is only very sensitive to changes around the midpoint of its input. Therefore, the limited sensitivity and saturation make the model need to adjust the weights more to improve performance. In contrast, ReLU (Rectified Linear Unit) is closer to the principle of bionics, has more efficient gradient descent and back-propagation, and a more simplified calculation process. The results of experiment have also proved that ReLU achieves better model performance. The BPNN’ parameters and their comparative experimental results are shown in Table 1:

**Table 1:** BPNNs’ parameters and experimental results comparison table.

Hidden layer structure	Maximum iterations	Weight optimizer	Activation function	Training time(s)	Weighted average of F1
3	300	L-BFGS	Sigmoid	18	0.85
18–18	300	SGD	ReLU	169	0.92
12-16-5	300	SGD	ReLU	228	0.93
12-16-5	300	Adam	ReLU	128	0.94
12-14-11-5	300	Adam	ReLU	202	0.94
12-10-10-5-5	300	Adam	ReLU	303	0.94
12-10-10-5-5-5	300	Adam	ReLU	190	0.92
12-16-5	300	Adam	Sigmoid	92	0.91
12-16-5	600	Adam	ReLU	131	0.94

Through the above analysis and comparison, the BPNN finally selected in this study contains three hidden layers. The number of nodes in each layer is 12, 16, and 5 respectively, the weight optimizer is Adam optimizer, the activation function is ReLU function, and the maximum number of iterations set to 300 times to prevent the program from falling into an infinite loop.

The article "Early warning of telecom enterprise customer churn based on ensemble learning" was published in 2023. Journal: PLoS One.

### Prediction model based on RF

#### Basic principle and structure of RF

RF is a Bagging (Bootstrap aggregating) classification model based on decision tree model. Take decision tree models as the base learners which are integrated into a strong learner through the strategies of parallel training and result integration. The specific structure is shown in Fig 2:

**Fig 2:** RF model’s structure.

RF performs self- sampling firstly. For a training data set of size ***N***, each time a subset of size ***M*** is selected from the data set by replacement sampling, and repeated ***K*** times to form ***K*** subsets. According to each subset, the dataset constructs ***K*** decision trees, so that each subtree analyzes the data from a different and one-sided perspective, and parallel learning does not affect each other’s results. Yu Sidong and Huang Xin in the airline customer churn analysis research believe that compared with ID3 and C4.5, the CART (Classification and Regression Trees) algorithm is more widely used and has significant effects, and prove that CART decision tree model does have a good effect on the prediction of customer churn [13]. Therefore, the node feature selection method of the decision subtree in this study is the CART model. The Gini index is used to select the optimal feature, and at the same time, the optimal binary value splitting point of the feature is determined. The construction steps of a binary decision tree from the root node are as follows:

(1) The Gini index of each feature is calculated for the training set ***D***. Suppose that each feature ***A*** contains ***k*** possible values ***a***_*i*_ (i = 1, 2, ……*k*), and divides ***D*** into two parts ***D***_***1***_ and ***D***_***2***_ according to the value of ***A*** is ***a***_*i*_ or not. The Gini index formula for A is shown in Eq (6):
$$Gini(A)=1-\sum_{i=1}^{k}p_{a_{i}}^{2}$$ (6)
  where *p*_*ai*_ is the probability of V(*A)* = *a*_*i*_.
(2) Among all features ***A*** and all their split points *a*_*i*_, the feature with the smallest Gini index and its corresponding split point are selected as the optimal feature and optimal split point. Then two child nodes are generated from the current node accordingly, and the training data sets are assigned to two child nodes by feature.
(3) Steps (1) and (2) are called recursively for two child nodes until the condition is met to stop the CART tree growth.

After all subtrees are constructed and the results are output, the RF will aggregate the results, use ***K*** models to predict separately, and then obtain the final prediction result by taking the average or majority classification result. For the binary classification problem studied in this paper, the final prediction result is usually obtained by majority-voting. The calculation process is shown in Eq (7):

$$h(S)=\frac{1}{M}\sum_{m=1}^{M}I(h_{m}(S_{m})=Y)$$ (7)

when ***h(S)*** is the final prediction result of RF, ***M*** is the subtree, ***I*** is the indicative function, ***h***_***m***_***(S***_***m***_***)*** is the single decision tree, and ***Y*** is the prediction result of the subtree.

The article "Early warning of telecom enterprise customer churn based on ensemble learning" was published in 2023. Journal: PLoS One.

In the study of predicting cardiovascular disease by Shinya Suzuki et al., the RF model predicts better than traditional logistic regression [14]. In the research on overdue prediction of provident fund loans, Hua Guangrong achieved an improved RF model with higher accuracy than XGBoost and traditional RF by adding threshold improvement [15]. Xu Jiaqing et al. realized a high-performance interconnection network congestion fault detection model based on RF, and the effect is better than the three algorithms, that is SVM, Naive Bayes, and Adaboost [16]. Wu Peiqi et al. also conducted a study on the identification of benign and malignant breast lesions, and found that the diagnostic accuracy of RF was higher than that of SVM and logistic regression models [17]. Regarding the Neural Network and Adaboost model related to this paper, Kristiawan Nugroho et al. proved that the accuracy of the RF model is higher than that of the neural network and Adaboost in the hate speech judgment study of the Twitter website [18].

In summary, in the field of machine learning and data analysis, RF has been adopted by a large number of research topics, and has generally achieved good results. It has high accuracy in various prediction problems, and in the actual application process, it is not easy to produce over-fitting because of its random sub-sample set and random feature selection. In addition, RF also has many advantages, such as strong anti-noise ability (noise refers to abnormal data), good at processing high-dimensional data with more features, strong universality and so on. Compared with the current various machine learning models, the training time is also very short, which is suitable for secondary integration as a base learner that can quickly draw accurate prediction conclusions. Therefore, this study chooses RF as one of the prediction models of customer churn.

The article "Early warning of telecom enterprise customer churn based on ensemble learning" was published in 2023. Journal: PLoS One.

#### RF model design and implementation

The basic parameters of the RF model are analyzed and set as following:

(1) The number of sub-trees—Usually the more the number of sub-trees, the better the effect of the model is. If the number of sub-trees is too small, it will lead to underfitting problem, but too many sub-trees will lead to training too long and accuracy not been improved, even overfitting problem. Because the number of features in the operator ’s customer data set is small, which is only 14, and there is no limit on the maximum feature usage of each subtree, the correlation of the generated RF subtrees is relatively high, and there is no need for too many subtrees to participate in the integration. The experimental results also show that 10 subtrees can achieve relatively stable and excellent prediction results. When the number of subtrees reaches 30, the comprehensive accuracy rate is the same, but the prediction accuracy rate for positive samples fluctuates between 94% and 95%. When it reaches 40, it is stable, and then increases to 100 will not change the results.
(2) Subtree generation algorithm—Because the ID3 algorithm is more classic, only the incremental information entropy is used to select the splitting features, and the features with a large number of values are preferred. Therefore, the CART algorithm uses the Gini index to avoid such defects. And unlike the ID3 algorithm to generate a multi-branch tree, the dichotomy of the CART algorithm also reduces the size of the decision tree and improves the efficiency of subtree generation. The results show that the indexes of the model based on Gini index and information entropy are the same, but the training speed of information entropy is slow, which proves that it is appropriate to use Gini index as the standard of subtree generation.

In addition, the minimum number of samples required for the re-division of internal nodes, the minimum number of samples required for the leaf nodes, the maximum depth of the subtree, the maximum feature usage and other parameters are mainly used in the study with a large number of samples. So there is no need to limit here, and experiments show that the prediction performance of the model decreases with the increase of its value. Each RF models’ parameters and comparative experimental results are shown in Table 2:

**Table 2:** RF models’ parameters and experimental results comparison table.

Number of sub-trees	Subtree generation algorithm	The minimum samples for redividing	Minimum samples in leaf node	Training time(s)	F1 value of Positive samples	Weighted average of F1
10	gini	2	1	5	0.94	0.97
30	gini	2	1	15	0.94~0.95	0.97
40	gini	2	1	20	0.95	0.97
100	gini	2	1	52	0.95	0.97
10	entropy	2	1	6	0.94	0.97
10	gini	30	1	4	0.93	0.96
10	gini	2	10	4	0.92	0.96
10	gini	2	1	3	0.89	0.94
10	gini	2	1	5	0.94	0.97
10	gini	2	1	5	0.94	0.97

Through the comparative analysis of the experimental results, the RF model adopted contains 40 sub-trees, the sub-tree is the CART binary decision tree generated by the Gini index, the minimum number of samples required for the re-division of internal nodes is 2, the minimum number of samples of leaf nodes is 1, and the maximum depth and maximum feature usage of the sub-tree are not limited.

The article "Early warning of telecom enterprise customer churn based on ensemble learning" was published in 2023. Journal: PLoS One.

### Prediction model based on Adaboost

#### Basic principle and structure of Adaboost

Adaboost is one of the successful representatives of Boosting ensemble algorithm. The basic idea is to add a weak classifier to each iterative training, and increase the weight of the samples that are misclassified in the last iteration. After reaching the maximum number of iterations ***N***, the ***N*** classifiers are used to comprehensively determine the final prediction result. The specific process is shown in Fig 3:

**Fig 3:** Adaboost model’s structure.

The steps of Adaboost algorithm are roughly divided into the following three parts:

(1) Initialize the weight of training data. Suppose the original data set T is represented as Formula (8):
$$T=\{(X_{1},Y_{1}),(X_{2},Y_{2}),(X_{3},Y_{3}),\ldots ,(X_{N},Y_{N})\}$$ (8)
  Where ***N*** is the number of all samples of the data set ***T***, and the ***N*** samples will be given the same weight value ***1/N***. The initial weight matrix ***D***_***1***_ is shown in Formula 9:
$$\left\{ \begin{array}{l} D_{1}=(w_{1,1},w_{1,2},\ldots ,w_{1,i})\\ w_{1,i}=\frac{1}{N} \end{array},i=1,2,\ldots ,N\right.$$ (9)
(2) Training base classifier. The number of iterations is ***m*** = 1, 2,……, M, the training set with the weight matrix ***D***_***m***_ is input and trained to obtain the base learner ***G***_***m***_**(*x*)**, and the classification error rate ***e***_***m***_ of ***G***_***m***_**(*x*)** to the data set is calculated. The calculation process is shown in Formula 10:
$$e_{m}=\sum_{i=1}^{N}w_{m,i}I(G_{m}(x_{i})\neq y_{i})$$ (10)
  In the training process, Adaboost changes the weight of samples and base learners to pay attention to samples with wrong classification and base learners with small errors. The weight of the base learner ***G***_***m***_**(*x*)** in the final strong learner ensemble is shown in Formula 11:
$$a_{m}=\frac{1}{2}\log\frac{1-e_{m}}{e_{m}}$$ (11)
  For sample weights, the updated dataset weight matrix is expressed as Eq 12:
$$D_{m+1}=(w_{m+1,1},w_{m+1,2},\ldots ,w_{m+1,i}),i=1,2,\ldots ,N$$ (12)
  The weight ***w***_***m+1***_ is updated as shown in Formula 13:
$$w_{m+1,i}=\frac{w_{m,i}}{Z_{m}}\exp(-\alpha_{m}y_{i}G_{m}(x_{i}))$$ (13)
  In order to ensure the probability distribution of the sample is 1, ***Z***_***m***_ is the normalization factor, and the expression is shown in Formula 14:
$$Z_{m}=\sum_{i=1}^{N}w_{mi}\exp(-\alpha_{m}y_{i}G_{m}(x_{i}))$$ (14)
(3) Base classifier integration—In the final classification ensemble function, the base classifier with small classification error rate will have a greater decisive effect on the final prediction result due to its larger weight. The strong learner ensemble strategy is shown in Formula 15:
$$F(x)=sign(\sum_{i=1}^{N}\alpha_{m}G_{m}(x))$$ (15)
  In the practical application process, Adaboost generally shows high classification accuracy, and it is not easy to produce over-fitting problems. Since the Adaboost algorithm only provides a framework, the specific base learner can be constructed by various methods, which has good flexibility and scalability, and pays more attention to the classification of errors in the iterative process, so that the training error decreases exponentially. Therefore, this study chooses Adaboost as one of the prediction models of customer churn.

The article "Early warning of telecom enterprise customer churn based on ensemble learning" was published in 2023. Journal: PLoS One.

#### Adaboost model design and implementation

The basic parameters of Adaboost model are analyzed respectively, and the following conclusions are drawn:

(1) Base learner—Adaboost is only an integrated algorithm of base learner. In the current large number of studies, the Adaboost model taking decision tree as base learner is the most widely used. In the study of loan default risk prediction, Li Zhaofei proved that Adaboost model based on decision tree is more accurate than traditional decision tree and logistic regression [19]. The Adaboost model based on single-layer CART decision tree is also used in the study of heavy vehicle rollover warning by Ju et al., and the prediction accuracy is much higher than the logistic regression model [20]. Ye Lin et al. also found that the Adaboost model based on decision tree has a higher diagnostic accuracy for breast cancer than GaussianNB and KNeighbors algorithms, reaching 96.49% [21]. Therefore, this chapter selects CART classification stump with depth of 1 as the base learner of Adaboost model.
(2) The number of iterations—Since the essence of the Adaboost model is to strengthen the learning and adjustment of the misclassified samples through continuous iterations, the algorithm must have enough iterations. However, too many iterations not only have no effect on the experimental results, but also lead to a doubling of the training time. Experiments show that when the number of iterations increased to 320 the indicators are the highest, and they do not continue to increase with the number of iterations increasing.
(3) Learning rate—The learning rate represents the gradient convergence speed of the algorithm. Too large will miss the optimal value, and too small will make the convergence speed slow. Since the learning rate is essentially similar to the black box parameter, it can only find the balance with the number of iterations by constantly trial. According to the experimental results, when the learning rate is 1.8, the extreme value is reached, and the larger or smaller will lead to the decrease of the prediction performance. When the learning rate is increased to 2, the indicators will show a cliff-like decline.
(4) Lifting criterion—The lifting criterion is judged according to the misclassification ratio, and the difference is mainly the measurement of the weight of the base learner. SAMME focuses on the misclassification samples of a single base learner based on the probability of sample prediction error, while SAMME.R judges the total misclassification ratio of samples based on all base learners, and pays more attention to the integrity of all base learners. The results show that although the SAMME.R method takes a little longer to train, it improves the prediction accuracy of positive samples by 1%. The Adaboost models’ parameters and the comparative experimental results are shown in Table 3:

**Table 3:** Adaboost models’ parameters and experimental results comparison.

Iteration times	Learning rate	Lifting criteria	Training time(s)	F1 value of positive samples	Weighted average of F1
50	1	SAMME.R	20	0.88	0.94
50	1	SAMME	18	0.87	0.93
300	1	SAMME.R	118	0.92	0.95
320	1	SAMME.R	125	0.92	0.96
400	1	SAMME.R	164	0.92	0.96
320	1.5	SAMME.R	125	0.93	0.96
320	1.8	SAMME.R	125	0.94	0.96
320	1.9	SAMME.R	124	0.93	0.96
320	2.0	SAMME.R	124	0.39	0.41

Through the comparative analysis of the above parameters, the final Adaboost model base learner is a CART decision stump with a depth of 1. The base learner has 320 self-boosting times and a learning rate of 1.8. The lifting criterion adopts SAMME.R that focuses on the overall error sample ratio.

The article "Early warning of telecom enterprise customer churn based on ensemble learning" was published in 2023. Journal: PLoS One.

### Prediction dual-ensemble model based on RF-Adaboost

#### Basic principle and structure of dual-ensemble model

According to the three classical machine learning models constructed above, it is not difficult to find that the base learner used by Adaboost is only a simple single-layer decision tree. Due to the poor performance of the base learner, it does not maximize the effect of Adaboost, nor does it take advantage of the strong scalability of Adaboost algorithm. The outstanding advantages of the RF selected are the shorter training time, the simpler training process and the more accurate prediction results, but it has lower recall rate. Therefore, other combination strategies can be introduced to make full use of this advantage, thus breaking through the performance bottleneck of the RF model.

In 2021, Ji Junhong et al. proposed a GSK-AdaBoost-RF model based on RF as the basic algorithm, combined with AdaBoost integration method and parameter optimization in the prediction of geological disasters-rock burst. Compared with the traditional RF model with the best effect before, the accuracy of rock burst prediction increased by 16.7% [22]. Therefore, considering that both RF and Adaboost model are in the bottleneck of rising prediction performance, this paper draws on previous research ideas and innovatively proposes the RF-Adaboost dual-ensemble model.

The structure of the RF-Adaboost is shown in Fig 4 following:

**Fig 4:** RF-Adaboost model’s structure.

RF-Adaboost dual-ensemble model refers to the secondary integration of several RF models as base learners through Adaboost ensemble strategy. In the previous content we can know that the RF belongs to the Bagging integration algorithm based on the decision tree, and the Adaboost belongs to the Boosting integration algorithm based on the decision tree. The RF-Adaboost essentially makes the two integration strategies work together, and the Bagging is continuously improved through the Boosting strategy to achieve the complementary advantages of time length and scalability, so as to give full play to the maximum effect of the two types of learning models of RF and Adaboost, and obtain more accurate prediction results for operator customer churn.

#### Dual-ensemble model design and implementation

The RF model has high accuracy, strong anti-overfitting ability and good anti-noise ability. However, when the number of decision trees in the forest is large, it has large space and time complexity. Adaboost model has high accuracy, simple structure of weak learner, and is easy to understand, but has poor anti-noise ability. Therefore, the two models with high accuracy and complementary advantages and disadvantages are considered to be combined to be a new strong model.

The Adaboost algorithm requires hundreds of iterations of the base learner, and the training time of a single base learner must be short enough. From the experimental results it can be seen that the model containing 10 subtrees and 40 subtrees has the very similar prediction accuracy rate, but there is a gap of 5 times in the training time. Therefore, the base learner of the dual ensemble model selects the 10 subtrees RF with a training time of only 5 seconds, rather than the 40 subtrees RF constructed in section RF model design and implementation.

The article "Early warning of telecom enterprise customer churn based on ensemble learning" was published in 2023. Journal: PLoS One.

For the outer Adaboost model, it is found through repeated experiments that all kinds of parameter values will not affect the final results of the double integrated model. Even when the learning rate is 2, the cliff-like decline of each index does not occur, but remains unchanged. Therefore, this study selected 50 iterations with short training time and the best 1.8 learning rate as the final parameters of the outer Adaboost model to maximize the efficiency and prediction performance of the model. The parameters and experimental results comparison of each RF-Adaboost models are shown in Table 4:

**Table 4:** The parameters and experimental results comparison of RF-Adaboost models.

Iteration times	Learning rate	Lifting criteria	Training time(s)	F1 value of positive samples	Weighted average of F1
50	1	SAMME.R	605	0.95	0.97
50	1	SAMME	605	0.95	0.97
300	1	SAMME.R	3607	0.95	0.97
50	1.8	SAMME.R	605	0.95	0.97
50	2.0	SAMME.R	604	0.95	0.97

### Comparison and analysis of model results

#### Evaluation indicators

The evaluation index used is calculated based on the confusion matrix of the preliminary evaluation index of binary classification prediction. In the binary classification problem, the final prediction results of the model are expressed by 1 and 0, namely positive and negative. The comparative analysis of the real value and the predicted value can be calculated by the True Positive, True Negative, False Positive, False Negative of the confusion matrix.

The specific structure of the confusion matrix is shown in Table 5:

**Table 5:** Confusion matrix.

Confusion Matrix		Real Value	
		Positive	Negative
Prediction Value	Positive	**TP**	**FP**
	Negative	**FN**	**TN**

Through the four basic indicators of the confusion matrix, the evaluation indicators can be extended and calculated. The following positive samples are taken as examples:

Precision—refers to the proportion of correctly predicted samples in all samples predicted by the model as positive. The formula is shown in Formula 16:

$$precision=\frac{TP}{TP+FP}$$ (16)

Recall rate—also known as sensitivity, refers to the proportion of correctly predicted samples in all samples that are actually positive. The formula is shown in Formula 17:

$$recall=\frac{TP}{TP+FN}$$ (17)

F1-score—is the combination index of precision rate and recall rate, where ***p*** represents precision rate and ***r*** represents recall rate, which can be considered as the comprehensive effect of the model. The formula is shown in Formula 18:

$$F1-score=\frac{2pr}{p+r}$$ (18)

The final model evaluation results include the accuracy rate, recall rate, F1 score, number of test samples of positive samples, the accuracy rate, recall rate, F1 score, number of test samples of negative samples, and the total sample weighted average of the above three indicators. The weight is the positive and negative ratio of the sample, reflecting the comprehensive performance of the model to predict all samples.

The article "Early warning of telecom enterprise customer churn based on ensemble learning" was published in 2023. Journal: PLoS One.

Since the research topic of this paper is the prediction of lost customers, in order to eliminate the impact of the prediction results of the non-lost samples that account for most of the proportion, more attention is paid to the prediction effect of the target samples. Among the above indicators, the recall rate of the positive samples is the most important indicator of the model effect evaluation.

(2) ROC curve—Receiver Operating Characteristic (ROC) curve, the abscissa is False Positive Rate (FPR), the ordinate is True Positive Rate (TPR), the calculation formula is shown in Formula 19, Formula 20:

$$FPR=\frac{FP}{FP+TN}$$ (19)

$$TPR=\frac{TP}{TP+FN}$$ (20)

The ROC curve obtains a pair of TPR and FPR values based on the performance of the model on the test samples, which is mapped to a point on the ROC plane. When the threshold is the largest, TPR = FPR = 0, corresponding to the origin of the image. When the threshold is minimum, TPR = FPR = 1, corresponding to the point (1, 1) in the upper right corner of the image. Therefore, by adjusting the classification threshold of the classifier, a corresponding point formed by several thresholds and a curve passing through (0, 0) and (1, 1) can be obtained, which is the ROC curve of the model. Since the test set is directly used as the threshold column in this study, the ROC curve consists of three points: (0, 0), (1, 1) and a single inflection point.

Among the evaluation indicators of the ROC curve model, the most commonly used is AUC (Area Under ROC Curve). The value of AUC is usually between 0.5 and 1.0 (0.5 is the area below the random classification curve). The larger the AUC value, the better the prediction performance of the model. For the ROC curve of the three-point production in this study, the most suitable observation method is to compare the distance from the inflection point to the (0, 1) point. Since the (0, 1) point represents that the judgment is a real case and there is no false positive sample point, that is, the prediction results are all correct, the closer the inflection point is to the upper left corner, the better the prediction effect of the model is.

The article "Early warning of telecom enterprise customer churn based on ensemble learning" was published in 2023. Journal: PLoS One.

#### Result comparison and analysis

This study mainly predicts the lost customers, that is, positive samples. Therefore, the comparative analysis of the performance of each model for the prediction indicators of positive samples is focused on. The recall rate of positive samples is the main reference index, and the precision rate of positive samples and F1 Score are secondary reference indexes. Based on the experimental data, Table 6 summarizes and compares the evaluation indexes of 9 machine learning models, including the BPNN, RF, Adaboost, RF-Adaboost double integrated model introduced above, the RF model constructed by reference [23], and the other four classical machine learning models-decision tree, naive Bayes, K-Nearest Neighbor, SVM.

**Table 6:** Comparison of model evaluation reports.

evaluating indicator	BPNN	RF	Adaboost	Decision Tree	Naive Bayes	KNN	SVM	RF-Adaboost	Reference [23]
**Positive Sample Recall Rate**	0.79	0.90	0.89	0.91	0.44	0.92	0.71	**0.93**	0.82
**Positive Sample Precision Rate**	0.97	**0.99**	0.98	0.89	0.60	0.84	0.94	**0.99**	0.98
**Positive Sample F1 Score**	0.87	0.95	0.94	0.90	0.51	0.88	0.81	**0.96**	0.89
**Negative Sample Recall Rate**	0.99	**1.00**	0.99	0.96	0.88	0.93	0.98	0.99	0.99
**Negative Sample Precision Rate**	0.92	0.96	0.96	0.96	0.80	**0.97**	0.89	**0.97**	0.93
**Negative Sample F1 Score**	0.96	**0.98**	**0.98**	0.96	0.84	0.95	0.94	**0.98**	0.96
**Weighted Avg Precision Rate**	0.94	0.97	0.97	0.94	0.74	0.93	0.91	**0.98**	0.95
**Weighted Avg Recall Rate**	0.94	0.97	0.96	0.94	0.76	0.93	0.90	**0.98**	0.95
**Weighted Avg F1 Score**	0.93	0.97	0.96	0.94	0.75	0.93	0.90	**0.98**	0.95

Take positive sample recall rate as the main reference index, the order of prediction performance from large to small is: RF-Adaboost > K-Nearest Neighbor > Decision Tree > RF > Adaboost > Reference [23] > BPNN > Support Vector Machine > Naive Bayes. The detailed comparison of the positive sample recall rate, precision rate and F1 Score of the nine models is shown in Fig 5.

**Fig 5:** Positive sample’s prediction indicators comparison of different models.

The comparison of experimental results shows that RF-Adaboost, KNN and decision tree perform well in the recall rate of positive samples, which is 93%, 92% and 91% respectively. RF-Adaboost, RF, Adaboost and Reference [23] perform well in the accuracy of positive samples, which is 99%, 99%, 98% and 98%, respectively. RF-Adaboost, RF and Adaboost perform well in the F1 value of positive samples, which is 96%, 95% and 94%, respectively. RF-Adaboost and K-nearest neighbor perform best in negative sample accuracy, both 97%; RF performs best in the negative sample recall rate, which is 100%; RF-Adaboost, RF and Adaboost performed well in the negative sample F1 value, which were 98%. RF-Adaboost, RF and Adaboost perform well in weighted average precision, weighted average recall and weighted average F1 value. Among them, the RF-Adaboost dual integration model has the best performance in 8 of the 9 indicators.

The article "Early warning of telecom enterprise customer churn based on ensemble learning" was published in 2023. Journal: PLoS One.

Compared with RF, the indicators of the RF-Adaboost are relatively close, but the positive sample recall rate is improved by 3%, indicating that the RF-Adaboost proposed in this paper has a significant improvement in the prediction ability of lost customers. In the longitudinal comparison of different studies, the recall rate of RF-Adaboost for positive samples increased by 10% on the basis of Reference [23], the precision rate increased by 1%, the F1 score increased by 6%, and the comprehensive weighted index increased by 3%.

It can also be seen from the experimental data that Naive Bayes performs the worst, with the recall rate even lower than 50% of the random binary classifier. The second worst is the KNN and SVM model. The former has a good recall rate (92%) but a general accuracy rate (84%), and the latter has an excellent accuracy rate (94%) but a low recall rate (71%). Both models have obvious prediction shortcomings, resulting in an integrated F1 value of less than 90%. The recall rate of the decision tree model for positive samples is 91%, and the precision rate is 89%. The prediction results are relatively better. Compared with RF-Adaboost model, the positive sample recall rate of decision tree is reduced by 2% and the precision rate is reduced by 10%.

In summary, the RF-Adaboost dual integration model is the best model of the nine models in terms of performance and comprehensive performance.

The ROC curves of the above nine machine learning models are compared as shown in Fig 6 following:

**Fig 6:** ROC curve comparison of models.

Through the comparison of nine ROC curves, it can also be seen intuitively that the inflection point of RF-Adaboost image is closer to the upper left corner than the other eight, which represents that RF-Adaboost has the highest prediction accuracy and recall rate among the nine models and the RF-Adaboost has the best prediction performance for operator customer churn.

For telecom operators with a large customer base, a 3% increase in the positive samples recall rate means that 300 wrong predictions are reduced from the 10,000 customer churn predictions. The fact is that the total number of customers currently held by domestic operators is hundreds of millions. Therefore, compared with the RF which has the second best prediction performance, the RF-Adaboost which improves the recall rate by 3% can save a lot of enterprise resources, achieve more accurate customer churn prediction, and facilitate telecom companies to implement more accurate customer retention strategies.

The article "Early warning of telecom enterprise customer churn based on ensemble learning" was published in 2023. Journal: PLoS One.

## Conclusion

Based on the current development trend of the telecommunications industry at home and abroad and the research status of operator customer churn, this paper adopts the gradually mature machine learning technology to predict the loss of operator customers based on. Eight machine learning models were constructed for training prediction-BPNN, RF, Adaboost, Decision Tree, naïve Bayes, KNN, SVM and the dual-ensemble model RF-Adaboost proposed in this paper. Comparative experiments are carried out for each model to select the optimal parameters, and the prediction results of the model are evaluated and displayed by the model evaluation index based on the confusion matrix and the ROC curve. The experimental results show that the RF-Adaboost has the highest positive sample recall rate for operator customer churn, reaching 93%, followed by KNN(92%)、Decision Tree(91%)、RF (90%), Adaboost (89%) and BPNN (79%). Compared with the reference [23], the recall rate of RF-Adaboost is also 10% higher, which proves the effectiveness of the proposed double integration model. Although various machine learning models are good at different fields and need to combine the advantages of different models in the research of a certain field, through comparative experiments and model integration, it is found that the overall effect of the models proposed in this paper is good, especially the RF-Adaboost double integration model, the prediction effect is best.

In the process of adjusting the parameters of the RF-Adaboost, it is found that the parameters of the model have no significant effect on the prediction performance. Therefore, future research on the project can focus on the attempt of other integrated models or the preprocessing part of the data set.

In the research of intrusion system behavior detection, by using SMOTE oversampling algorithm, RUS undersampling algorithm, random balance and other data processing operations in each iteration of Adaboost, the detection accuracy was higher than that in the preprocessing part [24]. The Adaboost model processed by SMOTE and RUS sampling algorithms performed better. Cheng Jianhua also constructed an ADmR-AdaboostSVM classification model based on SVM in the research of bond default warning [25]. ADASYN oversampling operation was carried out on the unbalanced data set, and the feature extraction mRMR method was introduced to screen the early warning indicators. Finally, the prediction result of 85% accuracy was achieved by the improved sampling Adaboost model. Therefore, in the future, further attempts and improvements can be made in data set processing. Various data processing algorithms, such as RUS undersampling, particle swarm optimization algorithm, K-means clustering algorithm, etc., which are widely used at present, can be selected and deeply integrated with the training process of machine learning model. Combined with previous research results, better data processing methods may be found through comparative experiments.

The article "Early warning of telecom enterprise customer churn based on ensemble learning" was published in 2023. Journal: PLoS One.

## Supporting information

S1 Data (ZIP)
